The article "Airway transplantation: a challenge for regenerative medicine" was published in 2013. Journal: Eur J Med Res.

# Airway transplantation: a challenge for regenerative medicine

**DOI:** 10.1186/2047-783X-18-25

**Published:** 2013-07-29

**Authors:** Emmanuel Martinod, Agathe Seguin, Dana M Radu, Guillaume Boddaert, Kader Chouahnia, Anne Fialaire-Legendre, Hervé Dutau, Nicolas Vénissac, Charles-Hugo Marquette, Christophe Baillard, Dominique Valeyre, Alain Carpentier, the FREnch Group for Airway Transplantation (FREGAT)

**Affiliations:** 1 Assistance Publique-Hôpitaux de Paris, Hôpitaux Universitaires Paris-Seine-Saint-Denis, Avicenne Hospital, Department of Thoracic and Vascular Surgery, Paris 13 University, Sorbonne Paris Cité, Faculty of Medicine SMBH, Bobigny, France; 2 Alain Carpentier Foundation, EA Laboratory for Biosurgical Research, Assistance Publique-Hôpitaux de Paris, George Pompidou European Hospital, Paris Descartes University, Paris, France; 3 Assistance Publique-Hôpitaux de Paris, Hôpitaux Universitaires Paris-Seine-Saint-Denis, Avicenne Hospital, Department of Oncology, Paris 13 University, Sorbonne Paris Cité, Faculty of Medicine SMBH, Bobigny, France; 4 Assistance Publique-Hôpitaux de Paris, Saint Antoine Hospital, EFS Ile de France, Tissue Bank, Paris, France; 5 Assistance Publique-Hôpitaux de Marseille, Thoracic Oncology, Pleural Diseases and Interventional Pulmonology Department, North University Hospital, Marseille, France; 6 CHU Nice, Pasteur Hospital, Department of Thoracic Surgery, Nice, France; 7 CHU Nice, Pasteur Hospital, Department of Pneumology, Nice, France; 8 Assistance Publique-Hôpitaux de Paris, Hôpitaux Universitaires Paris-Seine-Saint-Denis, Avicenne Hospital, Department of Anesthesiology and Intensive Care, Paris 13 University, Sorbonne Paris Cité, Faculty of Medicine SMBH, Bobigny, France; 9 Assistance Publique-Hôpitaux de Paris, Hôpitaux Universitaires Paris-Seine-Saint-Denis, Avicenne Hospital, Department of Pneumonology, Paris 13 University, Sorbonne Paris Cité, Faculty of Medicine SMBH, Bobigny, France

**Keywords:** Airway, Allograft, Aorta/aortic, Bronchial disease, Homograft, Lung cancer surgery, Tracheal disease, Tracheal surgery

## Abstract

After more than 50 years of research, airway transplantation remains a major challenge in the fields of thoracic surgery and regenerative medicine. Five principal types of tracheobronchial substitutes, including synthetic prostheses, bioprostheses, allografts, autografts and bioengineered conduits have been evaluated experimentally in numerous studies. However, none of these works have provided a standardized technique for the replacement of the airways. More recently, few clinical attempts have offered encouraging results with *ex vivo* or stem cell–based engineered airways and tracheal allografts implanted after heterotopic revascularization. In 1997, we proposed a novel approach: the use of aortic grafts as a biological matrix for extensive airway reconstruction. *In vivo* regeneration of epithelium and cartilage were demonstrated in animal models. This led to the first human applications using cryopreserved aortic allografts that present key advantages because they are available in tissue banks and do not require immunosuppressive therapy. Favorable results obtained in pioneering cases have to be confirmed in larger series of patients with extensive tracheobronchial diseases.

The article "Airway transplantation: a challenge for regenerative medicine" was published in 2013. Journal: Eur J Med Res.

## Review

Inhibition to tracheal surgery before 1960 was explained by difficulties related to perioperative ventilation, the poor healing capacity of cartilage and, finally, the “2-cm Belsey rule” stipulating that it was not possible to remove more than 2 cm of the trachea with primary reconstruction [1]. With the experimental and clinical studies stimulated over the past 50 years by Hermes C Grillo of Boston and some other surgeons around the world, all problems have been solved to provide a standardized approach to tracheal surgery [2]. In summary, using mobilization procedures, current surgical techniques permit the resection of approximately half of the adult trachea with reconstruction by primary anastomosis [3]. Proven methods are also available for laryngotracheal as well as carinal resection and reconstruction [4,5]. All problems have been solved, except one: the surgical treatment of extensive lesions where tracheal resection with primary anastomosis is not possible or is associated with a high rate of morbidity and mortality. As a result, patients with these lesions are only offered palliative care. To envision tracheal reconstruction after resection of extended lesions, we are in need of a tracheal substitute. Significant advances in medicine have allowed the successful replacement of complex organs. In contrast, attempts to replace the trachea, a rather simple conduit dedicated to the passage of air, have failed [6]. Thus, tracheal replacement remains today a great surgical and biological challenge.

### Airway transplantation: the five main methods of research

In 2004, the various tracheal substitutes and techniques of reconstruction were classified by Grillo into five categories: foreign materials, nonviable tissues, tracheal allotransplantation, autogenous tissues and tissue engineering [6]. The ideal airway substitute has to be a biocompatible rigid but flexible tube that should facilitate reepithelialization, integrate with adjacent tissues and be resistant to stenosis and bacterial colonization. Attempts to do this with the use of foreign materials led to chronic infection, airway obstruction, migration of the prosthesis, erosion into major blood vessels and proliferation of granulation tissue. Implantation of nonviable tissues–chemically treated, frozen or lyophilized–has been associated with poor functional results. Tracheal allotransplantation has also been disappointing because of complications of graft necrosis or stenosis. In addition, immunosuppressive therapy should not be prescribed for the treatment of a malignancy. Consequently, these approaches have increasingly been abandoned. Reconstructions with autogenous tissues such as skin, fascia lata, pericardium, costal cartilage, bladder, esophagus or bowel are complex procedures. They have led to unsatisfactory results, with the possible exception of muscle or cartilage flaps. Since the pioneering studies by Vacanti and colleagues [7,8], efforts have been made to induce the formation of cartilaginous tubes covered with epithelial cells using tissue-engineering techniques. At the time Grillo wrote his reference textbook, tracheal replacement using the tissue-engineered technique had not yet been applied to malignant tumors, as it required the use of the patient’s own cells and because several months were required to construct the graft. Reviews on airway transplantation have usually concluded that none of the proposed tracheal substitutes offer consistent results sufficient to consider a standardized approach [6,9,10].

The article "Airway transplantation: a challenge for regenerative medicine" was published in 2013. Journal: Eur J Med Res.

### Development of *ex vivo* tissue engineering

Since the publication of Grillo’s textbook, significant advances have been observed in the area of *ex vivo* tissue engineering based on the use of stem cells [11,12]. The modern area of stem cell research started effectively in the mid-20th century and permitted the definition of fundamental properties of stem cells, such as self-renewal, clonogenicity and multipotentiality. These developments have allowed identification and classification of stem cells from totipotent to pluripotent, multipotent and progenitor cells. They also have led to culture and differentiation of stem cells to consider their use in therapy and tissue engineering. The use of embryonic or tissue-specific adult stem cells has recently been proposed for the treatment of various human disorders. In addition, *ex vivo* tissue engineering has emerged as a possible solution for tissue reconstruction. This method requires cultivated human cells, which are seeded in scaffolds using artificial bioreactors before implantation of the engineered structures. In 2008, the team directed by Birchall in London reported the first case of tissue-engineered airway transplantation in a patient with post-tuberculosis end-stage bronchomalacia [13]. Recipient epithelial cells and mesenchymal stem cell–derived chondrocytes were cultivated and seeded onto a decellularized human donor trachea within an artificial bioreactor. The authors reported that favorable results were seen 4 months after implantation. This technique has some limitations, however because of the shortage of human tracheal donors. Furthermore, it cannot be used in cancer lesions, because the patient’s epithelial cells are needed and a few months are necessary to obtain the graft. In 2011, some members of Birchall’s initial group reported the use of a bioartificial nanocomposite instead of a decellularized human donor trachea [14]. The bioartificial nanocomposite was seeded with autologous bone marrow mononuclear cells onto an artificial bioreactor. This technique was performed in a first patient with recurrent extensive cancer. The authors observed stem cell homing and cell-mediated wound repair with extracellular matrix remodeling and neovascularization of the graft. Stem cell mobilization and apoptosis inhibition were due to boosting and growth factor administration [15]. The results were positive after 5 months of follow-up. In 2012, Elliott and colleagues reported the case of the first pediatric patient who had stem cell–based, tissue-engineered tracheal replacement, with encouraging results after 2 years of follow-up [16]. In 2010, Delaere and colleagues in Leuven reported a new surgical procedure performed in one patient with extensive post-traumatic stenosis [17]. While the patient was receiving immunosuppressive therapy, a tracheal allograft was wrapped in the recipient’s forearm fascia. The tracheal allograft was progressively revascularized and fully lined with donor respiratory epithelium and recipient buccal mucosa. After withdrawal of immunosuppressive therapy at 4 months, the tracheal allograft was moved to its anatomical position with an intact blood supply. Satisfactory results were obtained with a 1-year follow-up. In addition to the need for immunosuppressive therapy, problems related to this treatment modality are similar to those observed with *ex vivo* engineered airways.

The article "Airway transplantation: a challenge for regenerative medicine" was published in 2013. Journal: Eur J Med Res.

### Use of aortic matrix for airway transplantation

The complex approach of *ex vivo* tissue engineering has been unable to recreate functional regenerated tissues or organs in most attempts. Thus, some investigators have proposed the use of the human body as a natural bioreactor to achieve *in vivo* tissue engineering [18]. In 1997, we proposed a different approach to airway transplantation. During our preliminary work on tracheal replacement, we noticed that one structure had been ignored: the aorta. This biological structure has major advantages; it is a tubular conduit with a diameter similar to the trachea’s. Moreover, it is well-known for its solidity, elasticity and resistance to infection. On the other hand, it has a major disadvantage: the risk of collapse. However, this can be avoided by the use of a stent. Our work has been performed in successive steps using as tracheal substitutes aortic autografts, then fresh and cryopreserved allografts [19-25]. No complications occurred in the majority of animals during a maximum follow-up of 3 years. The macroscopic evaluation was very surprising. First, there was no stenosis in cases where a stent was inserted into the graft. Second, there was an unexpected tracheal regeneration, including epithelium and cartilage (Figures 1 and 2). This regenerative process was also observed after replacement of the carina. At the beginning of our experiments, we used a nitinol stent. Facing the regeneration of cartilage, we decided to remove the stent. It was impossible, however, because of major adhesions following the use of this type of stent. As a result, we placed a silicone stent into the graft. Removal was easy, and there were no clinical consequences. This showed that the regenerated cartilage was functional. Histological examinations showed a progressive regeneration of epithelium from an inflammatory tissue to a squamous, mixed and mucociliary epithelium. The phenomenon we observed was similar to that seen in the repair described by others after epithelium destruction. This is a well-documented process arising from basal and mucosal cells of the native trachea. At all intervals, we found residual elastic fibers from the aortic tissue. The inflammatory process was associated with reconstruction by fibroblasts secreting collagen. To discover whether cartilage came from aortic cells or from recipient cells, we decided in the six last animals in the allograft study to implant aorta from male sheep to trachea of female sheep and to search for *SRY* genes in the newly formed cartilage. Using a type 2 collagen marker, we demonstrated that newly formed structures within the aortic graft were indeed cartilage. PCR studies showed *SRY* amplification for male specimens but no amplification for female specimens or the newly formed cartilage. This clearly showed that newly formed cartilage originated not from aortic cells but from recipient cells. Today we know that this process did not come from aortic cells. Furthermore, chondrocytes cannot migrate, and newly formed cartilage was distant from the native trachea. These two points evidently refute the possibility of regeneration from the native cartilage. The last hypothesis is that regeneration came from mesenchymal cells, local cells or, most probably, circulating stem cells from bone marrow, as this has been demonstrated for the repair of other organs. This was recently confirmed by our group in a rabbit model [26]. Cryopreserved aortic allograft seems to be the better option in the view of human applications because of availability in tissue banks, permanent storage and no need for immunosuppression. We demonstrated that regeneration of a functional tissue could also be obtained after tracheal replacement with cryopreserved aortic allografts, in contrast to decellularized or glutaraldehyde-treated aortic grafts [25]. The regenerative process followed the same pattern as previously described for fresh allografts. These results were confirmed in a pig model as discussed by others [27-29]. We also demonstrated that an arterial allograft could be a valuable bronchial substitute with results similar to those obtained after tracheal replacement [30]. We theorized that airway healing after replacement with biological scaffolds was the consequence of a mixed phenomenon associating airway approximation and regeneration [31].

The article "Airway transplantation: a challenge for regenerative medicine" was published in 2013. Journal: Eur J Med Res.

**Figure 1:** Histologic examination of cryopreserved aortic allograft at 6 months (sheep model) showing regenerated airway epithelium (hematoxylin and eosin staining; original magnification ×2.5).

**Figure 2:** Histologic examination of cryopreserved aortic allograft at 2 months (sheep model) showing regenerated cartilage (hematoxylin and eosin staining; original magnification ×10).

### From experiments to first human cases

In 2005, a multicentric clinical program started in France to evaluate this new technique for extensive primary tracheal tumors. Aortic autograft was not used because of the risk. Fresh, then cryopreserved aortic grafts were evaluated in six patients with, in the majority of cases, adenoid cystic carcinoma [32,33]. Tracheal resection was extended to the carina in four patients, to the right upper lobe in one patient and to the left lung in one patient. Carinal reconstruction was performed in three patients. A silicone stent–supported aortic graft, fresh in two patients or cryopreserved in four, was used as a tracheal substitute. A pectoral muscle flap was created. No immunosuppressive therapy was given. Resection was complete in all patients but one. There was no postoperative mortality. However, postoperative morbidity was high, especially in the first patients. This was mainly due to problems with anastomosis and the stent or to infection. In long-term evaluation with a mean follow-up of 34 months, patient 1 died from metastatic disease at 45 months, patient 2 died from hemoptysis at 26 months, and the other four patients were alive and disease-free, three of whom had a full-time occupation. As observed in the experimental phase, the aortic graft was covered by continuous epithelium. However, only calcifications were observed. There was no identified regeneration of mature cartilage. A contraction of the aortic graft was also observed, as previously found in animal studies [31]. Asymptomatic fistulae between the graft and esophagus were seen in half of the patients. For all these reasons, a definitive removal of the stent was not proposed. Our experimental works led also to the first bronchial transplantation performed to avoid the high-risk procedure of pneumonectomy [34]. This operation was performed in a patient with large proximal lung cancer and with three factors predictive of postoperative mortality: age, right side and neoadjuvant chemotherapy. The first step consisted of complete resection of the lung cancer using intrapericardial upper bilobectomy with lymph node removal. Bronchial resection was performed from the first centimeter of the right main bronchus to the origin of the lower lobe bronchus because of extraluminal adhesions. After opening the pericardium, mobilization procedures were still limited by the stretching of the inferior pulmonary vein and kinking of the pulmonary artery. Reconstruction was performed using a cryopreserved aortic allograft from a certified tissue bank. A custom-made, fully covered, conical nitinol stent (Silmet; Novatech, La Ciotat, France) was inserted into the graft to prevent airway collapse. This stent was specially fabricated for this innovative procedure and for this patient. At the end of the operation, the sparing right lower lobe reexpanded normally, and there was no anastomotic leakage. No immunosuppressive therapy was given. In the postoperative course, we observed a supraventricular arrhythmia leading to mild pulmonary edema that resolved after 24 hours of standard medical therapy and right lower lobe atelectasis with bronchial colonization that required fiberoptic bronchoscopies in addition to antibiotic treatment. Chest tubes were removed at day 5, and the patient was discharged at day 16 with a normal CT scan showing a functional right lower lobe. Pathologic examinations confirmed radical surgical resection. After follow-up of 1 year, we concluded that the operation was feasible with no technical problems, that there was no major complication associated with this procedure during the postoperative period, that the reimplanted right lower lobe remained functional with no complications related to the stent or the cryopreserved aortic allograft, that pulmonary function after the operation remained largely superior to the third of the predicted value and, finally, that the health-related quality of life of the patient was preserved. A prospective phase 1 feasibility study is now in progress at our center (TRACHEOBRONCART Trial).

The article "Airway transplantation: a challenge for regenerative medicine" was published in 2013. Journal: Eur J Med Res.

## Conclusions

It is still unclear whether we are closer to the Holy Grail of airway transplantation with the use of cryopreserved aortic allografts. However, what we know is that this structure could have key advantages because it is a biologic structure available at tissue banks. In addition, this ideal matrix promoted *in vivo in situ* tissue engineering in animal models. Moreover, this matrix can be used for benign and cancerous lesions. The current difficulties are related to the delayed cartilage regeneration and the need for a permanent stent in human. This requires new studies to establish a standardized solution to the thus far unsolved problem of airway transplantation.

## Competing interests

The authors declare that they have no competing interests.

## Authors’ contributions

All authors drafted the manuscript. All authors read and approved the final manuscript.

## References

[B1] BelseyRResection and reconstruction of the intrathoracic tracheaBr J Surg19503820020510.1002/bjs.1800381500814791963

[B2] GrilloHCGrillo HCDevelopment of tracheal surgery: a historical reviewSurgery of the Trachea and Bronchi2004Hamilton, ON, Canada: BC Decker Inc136

[B3] GrilloHCGrillo HCTracheal reconstruction: anterior approach and extended resectionSurgery of the Trachea and Bronchi2004Hamilton, ON, Canada: BC Decker Inc517548

[B4] GrilloHCGrillo HCLaryngotracheal reconstructionSurgery of the Trachea and Bronchi2004Hamilton, ON, Canada: BC Decker Inc549568

[B5] GrilloHCGrillo HCCarinal reconstructionSurgery of the Trachea and Bronchi2004Hamilton, ON, Canada: BC Decker Inc599618

[B6] GrilloHCGrillo HCTracheal replacementSurgery of the Trachea and Bronchi2004Hamilton, ON, Canada: BC Decker Inc839854

[B7] VacantiCACimaLGRatkowskiDUptonJVacantiJPTissue engineered growth of new cartilage in the shape of a human ear using synthetic polymers seeded with chondrocytesMater Res Soc Symp Proc1992252367374

[B8] VacantiCAPaigeKTKimWSSakataJUptonJVacantiJPExperimental tracheal replacement using tissue-engineered cartilageJ Pediatr Surg19942920120510.1016/0022-3468(94)90318-28176592

[B9] StegerVHampelMTrickIMüllerMWallesTClinical tracheal replacement: transplantation, bioprostheses and artificial graftsExp Rev Med Dev2008560561210.1586/17434440.5.5.60518803471

[B10] MartinodESeguinARaduDMarquetteCHCarpentierA[Advances in tracheal surgery: are we close to finding the ideal tracheal substitute?] [in French]Rev Mal Respir20102755456410.1016/j.rmr.2010.04.00120610071

The article "Airway transplantation: a challenge for regenerative medicine" was published in 2013. Journal: Eur J Med Res.

[B11] MimeaultMHaukeRBatraSKStem cells a revolution in therapeutics: recent advances in stem cell biology and their therapeutic applications in regenerative medicine and cancer therapiesClin Pharmacol Ther20078225226410.1038/sj.clpt.610030117671448

[B12] DvirTTimkoBPKohaneDSLangerRNanotechnological strategies for engineering complex tissuesNat Nanotechnol2011613222115111010.1038/nnano.2010.246PMC4059057

[B13] MacchiariniPJungebluthPGoTAsnaghiMAReesLECoganTADodsonAMartorellJBelliniSParnigottoPPDickinsonSCHollanderAPManteroSConconiMTBirchallMAClinical transplantation of a tissue-engineered airwayLancet20083722023203010.1016/S0140-6736(08)61598-619022496

[B14] JungebluthPAliciEBaigueraSLe BlancKBlombergPBozókyBCrowleyCEinarssonOGrinnemoKHGudbjartssonTLe GuyaderSHenrikssonGHermansonOJutoJELeidnerBLiljaTLiskaJLueddeTLundinVMollGNilssonBRoderburgCStrömbladSSutluTTeixeiraAIWatzESeifalianAMacchiariniPTracheobronchial transplantation with a stem-cell-seeded bioartificial nanocomposite: a proof-of-concept studyLancet20113781997200410.1016/S0140-6736(11)61715-722119609

[B15] BaderAMacchiariniPMoving towards in situ tracheal regeneration: the bionic tissue engineered transplantation approachJ Cell Mol Med2010141877188910.1111/j.1582-4934.2010.01073.x20406329PMC3823270

[B16] ElliottMJDe CoppiPSpeggiorinSRoebuckDButlerCRSamuelECrowleyCMcLarenCFierensAVondrysDCochraneLJephsonCJanesSBeaumontNJCoganTBaderASeifalianAMHsuanJJLowdellMWBirchallMAStem-cell-based, tissue engineered tracheal replacement in a child: a 2-year follow-up studyLancet2012380994100010.1016/S0140-6736(12)60737-522841419PMC4487824

[B17] DelaerePVranckxJVerledenGDe LeynPVan RaemdonckDLeuven Tracheal Transplant GroupTracheal allotransplantation after withdrawal of immunosuppressive therapyN Engl J Med201036213814510.1056/NEJMoa081065320071703

[B18] BadylakSFNeremRMProgress in tissue engineering and regenerative medicineProc Natl Acad Sci USA20101073285328610.1073/pnas.100025610720181571PMC2840480

[B19] MartinodEAupècleBZegdiRFornesPAzorinJFabianiJNCarpentierA[Segmentary replacement of the trachea with an aortic autograft: the "trachea-aorta”] [in French]Presse Med199928163810544694

[B20] MartinodEZakineGFornesPZegdiRD’AudiffretAAupècleBGoussefNAzorinJChachquesJCFabianiJNCarpentierAMetaplastic transformation of an aortic autograft into a tracheal tissue: surgical implicationsLife Sci200032345546010.1016/s0764-4469(00)00150-510879293

[B21] MartinodEZegdiRZakineGAupecleBFornesPd’AudiffretAChachquesJCAzorinJCarpentierAA novel approach to tracheal replacement: the use of an aortic graftJ Thorac Cardiovasc Surg200112219719810.1067/mtc.2001.11434611436064

The article "Airway transplantation: a challenge for regenerative medicine" was published in 2013. Journal: Eur J Med Res.

[B22] MartinodESeguinAPfeutyKFornesPKambouchnerMAzorinJFCarpentierALong term evaluation of the replacement of the trachea with an autologous aortic graftAnn Thorac Surg2003751572157810.1016/S0003-4975(03)00120-612735581

[B23] MartinodESeguinAHolder-EspinasseMKambouchnerMDuterque-CoquillaudMAzorinJFCarpentierAFTracheal regeneration after tracheal replacement with an allogenic aortaAnn Thorac Surg20057994294910.1016/j.athoracsur.2004.08.03515734409

[B24] SeguinAMartinodEKambouchnerMCampoGODhotePBrunevalPAzorinJFCarpentierACarinal replacement with an aortic allograftAnn Thorac Surg2006811068107410.1016/j.athoracsur.2005.07.07916488724

[B25] SeguinARaduDHolder-EspinasseMBrunevalPFialaire-LegendreADuterque-CoquillaudMCarpentierAMartinodETracheal replacement with cryopreserved, decellularized, or glutaraldehyde-treated aortic allograftsAnn Thorac Surg20098786186710.1016/j.athoracsur.2008.11.03819231406

[B26] SeguinABaccariSHolder-EspinasseMBrunevalPCarpentierATaylorDAMartinodETracheal regeneration: evidence of bone marrow mesenchymal stem cell involvementJ Thorac Cardiovasc Surg201314512971304e210.1016/j.jtcvs.2012.09.07923111025

[B27] JaillardSHolder-EspinasseMHubertTCopinMCDuterque-CoquillaudMWurtzAMarquetteCHTracheal replacement by allogenic aorta in the pigChest20061301397140410.1378/chest.130.5.139717099016

[B28] MakrisDHolder-EspinasseMWurtzASeguinAHubertTJaillardSCopinMCJashariRDuterque-CoquillaudMMartinodEMarquetteCHTracheal replacement with cryopreserved allogenic aortaChest2010137606710.1378/chest.09-127519801581

[B29] TsukadaHErnstAGangadharanSAshikuSGarlandRLitmanovichDDeCampMTracheal replacement with a silicone-stented fresh aortic allograft in sheepAnn Thorac Surg20108925325810.1016/j.athoracsur.2009.09.00520103247

[B30] RaduDSeguinABrunevalPFialaire-LegendreACarpentierAMartinodEBronchial replacement with arterial allograftsAnn Thorac Surg20109025225810.1016/j.athoracsur.2010.03.07920609787

[B31] MartinodETracheal replacement with a bioabsorbable scaffold in sheep [invited commentary]Ann Thorac Surg2010901797179810.1016/j.athoracsur.2010.08.00121095312

[B32] WurtzAPorteHContiMDesbordesJCopinMCAzorinJMartinodEMarquetteCHTracheal replacement with aortic allograftsN Engl J Med20063551938194010.1056/NEJMc06633617079776

[B33] WurtzAPorteHContiMDussonCDesbordesJCopinMCMarquetteCHSurgical technique and results of tracheal and carinal replacement with aortic allografts for salivary gland-type carcinomaJ Thorac Cardiovasc Surg201014038739310.1016/j.jtcvs.2010.01.04320381819

[B34] MartinodERaduDMChouahniaKSeguinAFialaire-LegendreABrilletPYDestableMDSebbaneGBeloucifSValeyreDBaillardCCarpentierAHuman transplantation of a biologic airway substitute in conservative lung cancer surgeryAnn Thorac Surg20119183784210.1016/j.athoracsur.2010.11.01321353009

